# Optimization of Students' Performance Prediction through an Iterative Model of Frustration Severity

**DOI:** 10.1155/2022/3183492

**Published:** 2022-08-16

**Authors:** Sadique Ahmad, Najib Ben Aoun, Mohammed A. El Affendi, M. Shahid Anwar, Sidra Abbas, Ahmed A. Abd El Latif

**Affiliations:** ^1^EIAS Data Science and Blockchain Laboratory, College of Computer and Information Sciences, Prince Sultan University, Riyadh 11586, Saudi Arabia; ^2^Department of Computer Sciences, Bahria University, Islamabad, Karachi Campus, Pakistan; ^3^Department of Information Technology, College of Computer Science and Information Technology, Al-Baha University, Saudi Arabia; ^4^REGIM-Lab Research Groups in Intelligent Machines, National School of Engineers of Sfax (ENIS), University of Sfax, BP 1173, Sfax 3038, Tunisia; ^5^Department of Artificial Intelligence and Software, Gachon University, Seongnam-Si, Republic of Korea; ^6^Department of Computer Science, COMSATS University, Sahiwal, Pakistan; ^7^Department of Mathematics and Computer Science, Faculty of Science, Menoufia University, Al Minufiyah, Shebeen El-Kom 32511, Egypt

## Abstract

Recent articles reported a massive increase in frustration among weak students due to the outbreak of COVID-19 and Massive Open Online Courses (MOOCs). These students need to be evaluated to detect possible psychological counseling and extra attention. On the one hand, the literature reports many optimization techniques focusing on existing students' performance prediction systems. On the other hand, psychological works provide insights into massive research findings focusing on various students' emotions, including frustration. However, the synchronization among these contributions is still a black box, which delays the mathematical modeling of students' frustration. Also, the literature is still limited in using insights of psychology and assumption-based datasets to provide an in-house iterative procedure for modeling students' frustration severity. This paper proposes an optimization technique called the iterative model of frustration severity (IMFS) to explore the black box. It analyzes students' performance via two modules. First, frustration is divided into four outer layers. Second, the students' performance outcome is split into 34 inner layers. The prediction results are iteratively optimized under the umbrella of frustration severity layers through the outer and inner iterations. During validation, the IMFS achieves promising results with various evaluation measures.

## 1. Introduction

The outbreak of COVID-19 and E-learning with Massive Open Online Courses (MOOCs) introduced new challenges for weak students. They brought significant changes in students' lifestyles, academic teaching methodology, and performance evaluation procedures. COVID-19 has significantly increased students' frustration as they struggle to achieve excellent grades and good employment opportunities [1–3]. A student with high frustration severity is likely to perform poorly in academic activities, e.g., assignments, quizzes, workshops, and examinations [4]. Also, they made optimization of students' performance prediction systems more challenging. Such systems highlight at-risk students for psychological counseling and extra attention. Also, the prediction system needs optimized students' frustration severity modeling. Earlier studies show that distractions and frustration are the significant issues during an E-learning environment that negatively impact student engagement in the class [5]. Many research findings statistically correlated the outbreak of COVID-19 with the students' frustration severity [6]. Besides, institutions have given more liberty to the students and employees in their daily schedules. They have changed teaching and working culture to recover from the adverse influence of COVID-19 and frustration.

The current study splits earlier research contributions into two groups to provide a comprehensive picture of a few challenges, i.e., (1) psychology and data analysis findings and (2) students' performance prediction approaches. First, data analysis and psychological findings provide meaningful information and correlation between factors such as frustration, the COVID-19 pandemic, E-learning, and the performance evaluation of at-risk students [7–9]. Second, the prior students' performance prediction approaches used the psychological findings and data analysis contributions to optimize performance computation models [10–14]. These various groups of studies are still limited in obtaining an optimized students' performance prediction system based on insightful frustration severity modeling [15–19]. This paper proposes an iterative model of frustration severity (IMFS) to optimize the students' performance prediction system thoroughly.

It considers students' frustration severity with two main modules, i.e., (1) digitization and quantization and (2) frustration severity module. During the in-depth quantization and digitization, the students' scores are divided into thirty-four periodic outcomes (with a period of 0.3). It ensures the in-depth consideration of students' performance under the frustration severity layers. Second, the frustration severity is split into four layers (levels) to estimate students' scores iteratively. Furthermore, the proposed model has four main iterations and thirty-four sub-iterations to predict a single student's score. It performs 136 (34 × 4) iterations to optimize the prediction result in a single round during the prediction process. The experimental study reveals that IMFS performs significantly in terms of various accuracy measures, i.e., *F*1 score, precision, and recall.

The rest of the work depicts literature (Section 2), the proposed model, analysis, discussion, and conclusions.

## 2. Literature

Since the outbreak of COVID-19, the educational institutions were swapped to E-learning which brought significant changes in students' social and academic life, including weak and excellent ones [20]. The online classes, isolation, social distancing, and lockdowns considerably affected the students' attitudes. Also, educational institutions were active in overcoming the adverse impact of COVID-19 and frustration severity through significant changes in their policies [21]. They have relaxed the policies by giving more liberty to employees' working schedules and moving students to online classes. However, these precautions are insufficient in such an alarming situation in the future. Indeed, a system that can predict students' performance for further treatment and counseling of a particular at-risk student is needed [22]. Therefore, we need to work in two directions to optimize existing performance prediction systems. The first step includes data analysis findings that could correlate the factors that negatively and positively affect students' performance. The second step is to simulate (or provide a mathematical model) the correlation between students' characteristics, e.g., frustration, COVID-19 effects, performance, and so on.

### 2.1. Prior Analysis

COVID-19 and natural components of students' learning adversely influence students' performance 2^2^. It is common in students during intense learning environments. So far, the literature demonstrated that only informal qualitative work had been done on students' frustration and performance. A proper systematic process needs to analyze the relationship between frustrations, severity, and the adverse influence on students' future performance. The previous studies have various models that can be replicated to optimize the existing prediction systems [23–29]. Moreover, the instructor usually overcomes students' frustration via collaborative assignments and class activities to provide the best opportunities for learning [30]. Through these activities, students learn how to play in frustration and an intense learning situation. They can easily share their problems with classmates and learn better in offline mode with face-to-face interaction [31]. COVID-19 boosted the negative correlation between students' achievements and frustration severity. So, it is essential to predict students' performance and control the negative emotional impact in such an alarming situation [32]. Institutions that have transformed from offline to online are experiencing new challenges, such as technological illiteracy [33].

### 2.2. Prior Students' Performance Prediction Approaches

Many scholars analyzed students' achievements and published insightful data analysis [34–37]. However, very meager work has been done in simulating the relationship between students' emotions (frustration, stress, etc.) and performance. Also, the published studies have many black boxes introducing new challenges while optimizing the current prediction system. Thus, the dire need is to evaluate the insightful data analysis and other opportunities to extend existing prediction approaches. Also, we need to analyze the qualitative findings of psychological literature to predict and simulate the influence of emotional factors. Excellent academic achievements are only possible with excellent cognitive skills. Usually, cognitive skills are considered the ability to perform any activity that needs reasoning and problem solving, i.e., assignments, quizzes, and written examinations [38–40]. These skills evolve as students learn and forget. Effective educational policies need such systems to adapt to the dynamic nature of students' cognition. So, these challenges are the main sources of inspiration for the proposed iterative model of frustration severity (IMFS).

## 3. Preliminaries

The proposed model implements the Bayesian inference method (BIM) over different nodes. BIM achieves posterior probabilities (PPs) of the most probable score of a student. BIM is based on four basic probabilities, given by the following definitions, i.e., prior, conditional, joint, and PP of students' scores. The conditional probability in BIM is given by equation (1). It shows that the probability of event A gives event B. On the other hand, we need a joint probability for BIM to finalize the PP. A joint probability is given by equation (2).

(1) $$\begin{array}{c} P\left(A|B\right)=\frac{P\left(A\cap B\right)}{P\left(B\right)}, \end{array}$$

(2) $$\begin{array}{c} P\left(A\cap B\right)=P\left(A\right)\times P\left(B\right). \end{array}$$

## 4. Proposed Iterative Model of Frustration Severity

The focus of the current attempt is to predict the expected students' scores while simulating the nonlinear influence of frustration severity. Thus, the IMSF methodology split frustration into four severity layers (where *s*1 refers to the first layer and *s*4 refers to the fourth layer of severity). This division of frustration severity has initiated IMFS. Also, the students' performance outcomes (0.1 ≤ performanceoutcome ≤ 10) are divided into thirty-four outcomes. The in-depth quantization of students' performance has finalized the second section of the IMFS. The primary goal of these layers is to accurately predict students' scores while ensuring the computation of frustration severity influence. Moreover, the division of layers ensures significant prediction accuracy.

### 4.1. Probability Calculation at IMFS Layers

To predict students' performance, the current approach selects the most probable score (out of 34) while computing each outcome's PP and the severe effects of frustration. IMFS embedded a machine learning model called BIM to calculate the most probable outcome of IMFS. IMFS embedded a machine learning model called BIM to compute the most probable outcome of IMFS. The result showed that IMFS achieved significant accuracy with the embedded BIM. BIM is easy to be embedded for the PP calculation. Thus, the BIM calculation finalizes the third section of the IMFS (of frustration severity).

### 4.2. Architecture of the Proposed Model

The IMFS has four main umbrella iterations to estimate the PP of students' performance outcomes (with respect to frustration severities). Each iteration includes 34 sub-iterations, which produces a set of 34 performance outcome PPs. The resulting PP set is refined in the next iteration. So, the proposed IMFS iteratively produces the PP of students' scores while considering the adverse effects of frustration.

### 4.3. Posterior Probability Estimation

During the training process, we randomly initiated the prior probabilities of students' performance outcomes, i.e., Figure 1 shows nodes of IMFS, which calculate PP under the influence of frustration. It depicts that the PP of students' performance outcomes is iteratively computed in each layer of the IMFS. During prior probability distribution, a probability weight is assigned from the interval of [0, 1].

(3) $$\begin{array}{c} {\text{SP}}_{\text{prior}}=S\left({\text{PS}}_{i}\right), \end{array}$$

(4) $$\begin{array}{c} {\text{Sp}}_{\text{prior}}^{c}=P\left({\text{SP}}_{j}^{c}\right)=i-{\text{SP}}_{\text{prior}}. \end{array}$$

Equations (3) and (4) show mutually exclusive and collectively exhaustive events. Moreover, SP_prior_ reveals the weight of prior probabilities (prior = 1 to 34), while 1 − SP_prior_ depicts the probabilities of various events, also referred to as mutually exclusive events. So, the probability of the first outcome of students' performance is depicted by SP_prior_. Also, the remaining thirty-three outcomes' probabilities are represented by 1 − SP_prior_. If we summarize the probability distribution in simple words, we can say that the probability [0, 1] is split into two sets. The probability of the first set is represented by equation (3) and the second set of probabilities is illustrated by equation (4). These both probabilities are mutually exclusive and collectively exhaustive. Furthermore, SP_prior_^*c*^ shows the probability of students' scores (where prior = 1 to 34) and SP_prior_^*c*^ illustrates the summation of thirty-three outcomes' probabilities. Additionally, the IMFS achieves the prior probabilities of frustration layers, which are shown by sev_prior_ (where prior = 1 to 4). Such probabilities are achieved for the computation of different students' score probabilities (joint and conditional).

(5) $$\begin{array}{c} {\text{PS}}_{cp}=P\left(sev_{k}|sp_{i}\right)=\frac{{\text{PS}}_{\text{prior}}\times sev_{\text{prior}}}{{\text{SP}}_{\text{prior}}}, \end{array}$$

(6) $$\begin{array}{c} {\text{PS}}_{m}^{c}=P\left(sev_{k}|{\text{PS}}_{i}^{c}\right)=\frac{1-{\text{PS}}_{\text{prior}}\times sev_{\text{prior}}}{1-{\text{PS}}_{\text{prior}}}. \end{array}$$

Equations (5) and (6) compute the conditional probabilities of students' performance, which are demonstrated by PS_*cp*_ and PS_*m*_^*c*^. Moreover, *cp* and *m* show various iterations for the computation of conditional probabilities. On the one hand, SP_prior_and 1−SP_prior_ illustrate the single frustration severity layers (also referred to as prior probabilities), and on the other hand sev_*k*_ depicts the remaining 4 layers of severity (where *k* = 1 to 4). Finally, SP_prior_^*c*^ depicts students' performance. In every computation round of *m*, the frustration probability (conditional) is analyzed. Also, *p* and *m* illustrated 68 iterations (sub-iterations) in each round of *p*.

(7) $$\begin{array}{c} {\text{SP}}_{{\text{joint}}_{xy}}=P\left({\text{sev}}_{k},sp_{i}\right)=\left({\text{SP}}_{\text{prior}}\right)\times \left({\text{SP}}_{cp}\right), \end{array}$$

(8) $$\begin{array}{c} {\text{SP}}_{{\text{joint}}_{\text{s}}^{c}}=P\left({\text{sev}}_{k},sp_{i}^{c}\right)=\left(1-{\text{SP}}_{\text{prior}}\right)\times \left({\text{SP}}_{m}^{c}\right), \end{array}$$

(9) $$\begin{array}{c} {\text{SP}}_{{\text{post}}_{mn}}=P\left(sp_{i}|sev_{k}=\frac{{\text{SP}}_{{\text{joint}}_{xy}}}{{\text{SP}}_{{\text{joint}}_{xy}}+{\text{SP}}_{{\text{joint}}_{s}^{c}}}|.\right. \end{array}$$

In equations (7) and (8), the variables SP_joint_*xy*__ and SP_joint_*s*_^*c*^_ represent the probability (joint) of students' outcome and the four layers of frustration, respectively. *xy* and *s* depict two rounds of iterations. The iterative model of frustration severity needs various types of probabilities to compute the final PP. In equation (9), the variable SP_post_*mn*__ shows the final probabilities of students' performance, also referred to as PP. Also, the range of *m* = 1 to 4 and *n* = 1 to 34. IMFS has four iterations for severity, while in each round of iteration, IMFS has thirty-four sub-iterations. Also, it should be noted that the obtained PP is considered before the next round of iteration. Every round of iteration produces a refined set of probabilities. Finally, IMFS chooses the most probable outcome of students' performance.

Algorithm 1 illustrates the iterative procedure of the proposed IMFS. As an input, it takes three sets of data; (1) sev consists of the information about frustration severity layers (*F*1 to *F*4), and (2) sp1 and sp2 consist of 34 prior probabilities of students' performance. The first loop initiates the principal iterations in which *i* chooses severity from sev (one by one). Furthermore, the algorithm starts an inner loop for the element of sp1. So, the variable *j* selects each element from sp1 (34 elements one by one) and calculates its PP under the influence of frustration severity. Each sub-iteration of the nested loop produces a PP of *J* with respect to the selected frustration severity (*i*). These PPs are achieved using equations (3)–(7). At the end of each step of the inner loop, the prior probability of a student's score is replaced by the PP of *j* of sp1. Thus, this process continues until the PP of the 34th performance outcome is calculated. The probabilities of 34 outcomes are re-estimated under the influence of four severity layers. Eventually, the first loop produces a set of refined PP.

Furthermore, Algorithm 1 consists of another module that compares the estimated values with actual values of students' performance outcomes, i.e., calculates prediction loss by (PL = (Actual − Measured)). This process evaluates the final PP of a student's performance outcome to enhance the accuracy of the proposed model. It compares the actual score with the most probable student's score (out of 34 PPs).

### 4.4. Statistical Algebraic Model for IMFS

The IMFS mathematically models the relationship among different frustration levels during various cognitive tasks, such as assignments, quizzes, final examinations, class activities, and group assignments. The following module shows the mathematical modulation of the proposed IMFS.

(10) $$\begin{array}{c} Fsev1^{k+1}=\text{SP}.Fsev1^{k}, \end{array}$$

(11) $$\begin{array}{c} Fsev2^{k+1}=\text{SP}.Fsev1^{k+1}, \end{array}$$

(12) $$\begin{array}{c} Fsev3^{k+1}=\text{SP}.Fsev1^{k+1}+\text{SP}.Fsev2^{k+1}, \end{array}$$

(13) $$\begin{array}{c} Fsev4^{k+1}=\text{SP}.Fsev1^{k+1}+\text{SP}.Fsev2^{k+1}+Fsev3^{k+1}. \end{array}$$

Equations (10)–(13) reveal the iterative correlation between frustration severity (*F*sev1 to *F*sev4) and students' expected score SP. Equation (10) shows SP under the umbrella of *F*sev1, and equation (11) reflects the accumulative effects of *F*sev1 and *F*sev2 on SP. Similarly, equation (12) shows the students' performance under the influence of accumulative influence of *F*sev1, *F*sev2, and *F*sev3 while equation (13) depicts the final value of students' performance (SP) under the umbrella of accumulative impact of four levels of frustration severity (*F*sev1, *F*sev2, *F*sev3, and *F*sev4).

### 4.5. Proof of Existence through Gauss–Seidel Method

The information in equations (10) to (13) is expressed in the Gauss–Seidel method using the following matrix.

(14) $$\begin{array}{c} \left[\begin{array}{c} F\text{sev}1^{k+1}\\ F\text{sev}2^{k+1}\\ F\text{sev}3^{k+1}\\ F\text{sev}4^{k+1} \end{array}\right]=\left[\begin{array}{cccc} SP & 0 & 0 & 0\\ 0 & SP & 0 & 0\\ 0 & SP & SP & 0\\ 0 & SP & SP & SP \end{array}\right]X\left[\begin{array}{c} F\text{sev}1^{k}\\ F\text{sev}1^{k+1}\\ F\text{sev}2^{k+1}\\ F\text{sev}3^{k+1} \end{array}\right], \end{array}$$

where *A* is the coefficient matrix representing students' scores while *B* is called augmented matrix.

Furthermore, the existence and uniqueness of such system are derived as

(15) $$\begin{array}{c} X=\text{AB}. \end{array}$$

Let *x* ∈ *R*+4 and $\bar{x}\in R+4$; then, we have the following equation.

(16) $$\begin{array}{c} \left\|x-\bar{x}\right\|=\left\|AB-A\bar{B}\right\|\\ =\left\|A\left(B-\bar{B}\right)\right\|\\ \leq \left\|A\right\|\left\|B-\bar{B}\right\|. \end{array}$$

Lastly, we have achieved ‖*A*‖ ≤ 1. It shows that system (1) has unique solution.

## 5. IMFS Prediction Result

The proposed approach was evaluated during the experiment using state-of-the-art measures such as precision, recall, accuracy, and *F*1 score. It automated the association between students' performance and frustration. Thus, the empirical result section is split into the following sections to evaluate the accuracy.

### 5.1. Data Collection Process

The proposed IMFS was analyzed with a students' score dataset during the experiment. This particular dataset is a new version of the dataset, which was collected during an interview [41].

#### 5.1.1. Population and Sampling

The data were collected in seven universities around different provinces of Pakistan. The particular universities are given below.

  Bahria University Karachi Campus.
  Bannu University of Science and Technology.
  Bacha Khan University Peshawar.
  Iqra University Karachi.
  Lakki University of Science and Technology.
  Information Technology University, Lahore.
  Institute of Management Sciences Peshawar.

The selections of universities and computer science (CS) departments are based on a convenience-based sampling technique. The participants from these universities, especially the CS department, were easily available. We have ensured a qualitative data collection process by selecting CS students for the experiment. The preparations for multiple CS-related quizzes under various frustration severity impacts were comparatively easy. So, the convenience-based sampling technique has ensured accurate information about the frustration severity. The study follows Yamane's (1967) standard to select enough samples from the targeted population. The Yamane formula for sampling is given below.

(17) $$\begin{array}{c} n=\frac{N}{1+N{\left(e\right)}^{2}}. \end{array}$$

According to the Yamane sampling formula (using population), the minimum sample size is 15700; however, we have oversampled the data up to 20000 to ensure the Yamane standard.

#### 5.1.2. Data Collection Methodology

We conducted 21 prank-based interviews in the institutions mentioned above to collect enough qualitative students' score data. Students were frustrated by negatively commenting on their performance. Such comments were made by the concerned teacher of the course in different universities. A student can be frustrated by negative comments on his future grades, performance, job opportunity, and family attributes [42]. Also, state-of-the-art findings were used to frustrate these students during the interview. Students' performances were evaluated on course-related quizzes. Psychological literature-based tactics were used to discourage the participants [43–49]. Also, we have developed various quizzes to assess the students' performance in different frustration severity. The performance outcome in the test depends on different factors, such as the amount of time taken during the test, their mistakes, and the logic of the solution. After the test, the particular student was informed about the nature of the ongoing experiment to sign the consent. The frustration severity was ensured via participants' self-assessment basis. We have assessed the performance of 451 students. So, 1804 samples were collected. To efficiently train IMFS, we oversampled the dataset to 20000 records based on psychological findings and theoretical data analysis contributions. Such assumption-based datasets pave the way for efficient training and testing of a deep model. Moreover, the correlation between different levels of frustration severity is highlighted by the Pearson correlation in Table 1, which is self-explanatory with Pearson correlation values and confidence intervals.

### 5.2. Training of IMFS

The training process was initiated with 10-fold cross-validations. Also, the study has five partitions of students' score outcomes, such as very low performance (at-risk students), low (still at-risk), average performance, good, and excellent (with outstanding performance). The IMFS achieved significant performance in terms of ten-fold cross-validation processes. Furthermore, 150 distinct tests were performed using ten samples of data. So, training and testing were carried out on various pairs (i.e., 90% training set and 10% test set). This section achieved a final set of prior probabilities [33] during IMFS training.

### 5.3. IMFS Prediction Assessment

The performance outcomes are distributed into five different partitions to show the performance results. On the one hand, the first four partitions consist of 28 students' score outcomes. On the other hand, the last partition consists of six score outcomes. Moreover, the study divided the performance range into various intervals, which are demonstrated as follows:

  (0.1 ≤ *SP* ≤ 1.9) as *P*I
  (2.2 ≤ *SP* ≤ 4) as *P*2
  (4.3 ≤ *SP* ≤ 6.1) as *P*3
  (6.4 ≤ *SP* ≤ 8.2) as *P*4
  (8.5 ≤ *SP* ≤ 10) as *P*5

Here, SP means students' performance. During the experiment, the PP of each partition is evaluated separately, i.e., PPs of the five partitions are estimated using the severity layer umbrella. During the method validation, we selected five random data samples. Each sample consists of thirty values. The IMFS receives a set of thirty-four probabilities along with the highest probability. In addition, the performance of IMFS was assessed with various validation models, such as recall, *F*1 score, and precision, while the training and testing have true positive, true negative, false negative, and false positive, represented by the following variables.

(18) $$\begin{array}{c} \text{Accuracy}=\frac{\sum_{i=1}^{4}\left({\text{TP}}_{i}\right)}{\sum_{i=1}^{4}\left({\text{TP}}_{i}+{\text{FP}}_{i}+{\text{TN}}_{i}+{\text{FN}}_{i}\right)}. \end{array}$$

The prediction results of IMFS (with P1 partition) are illustrated in Figure 2. The PP is shown in a red line graph depicting the actual PP of students' performance outcomes. The prior probabilities of the proposed technique are described in Table 2, working as coefficients to obtain the PP of the given inputs (frustration severity). To achieve the accuracy for *P*1, we have used equation (10) for performance calculation (where *i* = 1 to 5). TP denotes true positive, FP reveals false positive, TN represents true negative, and the FN manifests a false negative of the model. The list of state-of-the-art performance measures is given in Table 3. Eventually, the IMFS obtained significant performance in terms of validation models.

(19) $$\begin{array}{c} \text{Precision}=\frac{{\text{TP}}_{i}}{{\text{TP}}_{i}+\sum_{i=1}^{3}\left({\text{FP}}_{i}\right)}. \end{array}$$

Equation (11) measures the accuracy of students' performance outcome as a precision measurement. The parameters of equation (11) are explained earlier. The IMFS has received an excellent precision value for P1, i.e., see Table 3. Moreover, the recall measure (equation (12)) is used to calculate the accuracy of the proposed technique. Resultantly, the IMFS achieved a significant accuracy in terms of recall measure for P1, i.e., see Table 3.

(20) $$\begin{array}{c} \text{Recall}=\frac{{\text{TP}}_{i}}{{\text{TP}}_{i}+\sum_{i=1}^{3}\left({\text{FN}}_{i}\right)},\\ F1=2\times \frac{\text{precision }\times \text{recall}}{\text{precision }\times \text{recall}}. \end{array}$$

The proposed model achieved a significant result via the *F*1 score illustrated by equation (13), i.e., *F*1 scores in Table 3 and Figure 3. The red graph depicts predicted values, while the blue graph represents the original values of students' performance. The empirical analyses demonstrated significant results in every dataset partition. In addition, Figure 4 shows the accuracy of IMFS in *P*3 (partition three). The results have shown that the IMFS thoroughly simulated the correlation between frustration severity and *P*3. Also, the study examined the performance of IMFS (in terms of the validation measures as mentioned earlier) to validate its preciseness. So, it performed satisfactorily in different validation measures (see results in Table 3).  Figure 5 shows the result of IMFS for *P*4 (partition four), which depicted significant accuracy in terms of precision, recall, *F*1, and accuracy measures. Also, in Table 3, the study demonstrated the performance of IMFS for *P*4. Lastly, IMFS was thoroughly investigated in terms of *P*5 partition (prediction results are shown in Figure 6). On the one hand, the red graph illustrates the predicted values, while on the other hand, the blue graph shows original values of the students' scores. The proposed IMFS has iteratively modulated the nonlinear links among partition five and the severity of frustration. The result via validation models depicted significant results in terms of different parameters (for more information, see Table 3).

### 5.4. Assessment of the Most Probable Outcome of Students' Performance

The thirty-four outcomes of students' scores are split into five partitions to validate the proposed iterative model, i.e., very low, low, average, good, and finally, excellent performance outcome, as illustrated earlier. The technique separately simulated the relationship between frustration severity and students' scores during the second experiment. Also, each partition of students' scores has a probability interval [0, 1] distributed between seven outcomes. These particular distributions depend on the prior probabilities of students' performance outcomes. Before the prediction experiment, we hypothesized the relationship between students' performance and frustration severity. According to the hypothesis, the PP of the first three partitions (*P*1, *P*2, and *P*3) must be increased with severity. In comparison, the PP of the last two partitions (*P*4 and *P*5) might be decreased with an inevitable increase in frustration severity. The technique has achieved excellent prediction accuracy on students' datasets. These results illustrated that the PPs of the first three partitions (*P*1 to *P*3) are increasing under the intense influence of frustration severity. Figures 7–9 show *P*1 (very low), *P*2 (low), and *P*3 (average) students' scores, respectively. The increased rate in PP of P1 (Figure 7) is comparatively higher than P2 (Figure 8).

On the one hand, Figure 9 demonstrates that an increase in PP of *P*3 is comparatively higher than the increase in PP of *P*2. The first three partitions have revealed an increase in students' score probabilities under the influence of the four layers (*s*1 to *s*4). On the other hand, we have investigated the prediction results of the last two partitions (good = *P*4 and excellent = *P*5), which are shown in Figures 10 and 11. These two partitions' PPs are decreasing because frustration severity layers thoroughly influence *P*4 and *P*5 partitions. Also, the decrease rate of PP in *P*5 (Figure 11) is higher than that in *P*4 (Figure 10). These surprising results depicted that the proposed approach efficiently predicted the expected performance of students during cognitive tasks.

### 5.5. Comparative Analysis

As it can be seen from Table 4, the proposed IMFS is compared with three prior studies based on 11 significant features. They highlighted many technical challenges and efforts toward optimizing students' performance prediction systems; however, they could not achieve the 11 essential features mentioned in Table 4.

#### 5.5.1. Relevant Factor-Based Comparison

Earlier studies are saturated with many contributions that correlate students' performance with different levels of frustration severity (see section literature review). Also, state-of-the-art methods are insufficient to compute the adverse influence of frustration severity. As far as we know, the literature lacks algorithms that quantize frustration severity into multiple layers. It also lacks in splitting students' scores into thirty-four components to compute performance under the umbrella of the adverse impact of frustration severity. The quantization of performance outcomes and frustration severity is illustrated in Table 3.

#### 5.5.2. Iterative Prediction

The related work focused on student interaction with LMS, academic scores, and different family attributes; however, an optimized educational model is needed to mathematically model the frustration severity. So, the proposed IMFS computes students' performance under the umbrella of frustration severity clusters. Also, it addresses various challenges, such as optimization of prediction results with four outer layers and thirty-four inner layers. The current study optimizes students' performance prediction with in-depth frustration severity layers. The proposed system was trained and validated on an assumption-based and real-world dataset. These data were collected from seven different institutions to consider the additional demographic background data. Later, the dataset was extended based on psychological findings and theoretical data analysis discoveries. Nevertheless, the dataset used by state-of-the-art techniques is comparatively not sufficient for frustration severity challenges.

## 6. Discussion

Students' performance prediction has emerged as an exciting domain for many cognitive computing researchers and education-focused scientists. It has massive applications for critical cognitive tasks, such as performance prediction during students' class activities, written examinations, and quizzes. The study illustrated earlier that frustration severity continuously declines the performance of students. Therefore, it proposed an optimization method called the iterative model of frustration severity (IMFS) to predict students' scores while mathematically modeling the adverse influence of frustration severity. It has manipulated the nonlinear statistical relationship between the students' performance and frustration severity. This network consists of two main modules. First, frustration severity is split into four layers (*s*1 to *s*4). Second, the study digitized and quantized students' performance outcomes with a unique range (0.1 ≤ StudentPerformance ≤ 10) to ensure prediction accuracy. Also, the range of students' scores was split into 34 periodic discrete outcomes (with a period of 0.3). It manifests that the IMFS has two sets of layers, i.e., outer layers (frustration severities *s*1 to *s*4) and inner layers (34 layers of students' performance outcomes). During the prediction process, the first outer layer of the network produces a set of 34 unique posterior probabilities using equations (1)–(7). These posterior probabilities are optimized in the remaining three layers of frustration severity. Hence, the model produces an optimized set of posterior probabilities in each layer. Finally, the IMFS predicts students' performance by picking the score with the highest posterior probability. The proposed IMFS was tested on the students' scores dataset, which produced a significant accuracy in terms of various measures (results are presented in Table 3). Also, all the important abbreviations are shown in Table 5 and the parameter values of prior probabilities are depicted in Table 5.

The proposed model solves three challenges with the iterative procedure but also reports a few limitations. First, the proposed IMFS is instead a journey than a destination; therefore, the main loophole is the lack of extensive comparison based on prediction accuracy. Such comparison is planned in the future work (see Table 4 for novelty). Second, we have yet to perform extensive empirical tests using extended assumption-based and real-world datasets to ensure prediction accuracy. We also plan to add comprehensive quantization modules to optimize students' performance prediction process. Such a module will pave the way to assess the influence of other emotional attributes, such as various levels of frustration severity (instead of only four), depression, stress, and anxiety. Third, the severe effects of frustration are yet to be investigated by thoroughly examining the existing psychological work. Also, the study needs to explore the factors such as frustration and frustration severity by electroencephalography (EEG) because an individual's emotional status is always sensitive to the aforementioned emotional attributes. In addition, the following statement should be noted for future consideration.

  A series of experiments were conducted to validate the network's performance, and finally, we have chosen the average prediction results (i.e., see Table 3).
  The proposed model can produce different results in achieving different sets of prior probabilities for the intervals of students' scores and frustration severities.
  The performance outcomes are partitioned into five groups (*P*1 to *P*5) due to the nonlinear statistical correlation between students' performance and frustration severity; however, in future work, the study will simulate the relationship between frustration severity and each outcome of students' scores.

## 7. Conclusions

In this paper, we presented an iterative model of frustration severity (IMFS) to optimize the prediction of students' performance while modeling the influence of frustration severity. The IMFS has three main contributions. First, the student frustration severity was divided into four outer layers (*s*1, *s*2, *s*3, and *s*4) to model the severity influence. Second, the study divided the range of students' scores into thirty-four discrete periodic outcomes (periodic distance = 0.3), forming the IMFS inner layers. Third, it predicted students' performance with the two sets of layers. Finally, the IMFS was evaluated on students' score datasets. It achieved significant performance in terms of various accuracy measures, i.e., *F*1 score, precision, and recall.

## Figures and Tables

**Figure 1:** Framework of iterative model of frustration severity. SP shows students' performance outcomes and BIM stands for Bayesian inference method.

**Figure 2:** The prediction accuracy of IMFS in *P*1.

**Figure 3:** IMFS performance in *P*2.

**Figure 4:** The performance of IMFS in *P*3.

**Figure 5:** IMFS in *P*4.

**Figure 6:** The IMFS performance in *P*5.

**Figure 7:** The posterior probabilities of *P*1 (very low performance outcomes).

**Figure 8:** The probabilities of *P*2 are evolving with a change in frustration severity.

**Figure 9:** An increase in probabilities of *P*3 with respect to severity.

**Figure 10:** The posterior probabilities of *P*4.

**Figure 11:** The probabilities of *P*5 are decreasing due to the profound effect of severities.

**Algorithm 1:** Students' performance prediction process.

**Table 1:** Pearson correlations.

	Severity 1	Severity 2	Severity 3	Severity 4
Severity 1: Pearson correlation	1			
Severity 2: Pearson correlation	0.425^*∗∗*^	1		
Severity 3: Pearson correlation	0.373^*∗∗*^	0.450^*∗∗*^	1	
Severity 4:Pearson correlation	0.265^*∗*^	0.297^*∗*^	0.508^*∗∗*^	1

^*∗∗*^Correlation is significant at 0.01 level (2-tailed). ^*∗*^Correlation is significant at 0.05 level (2-tailed).

**Table 2:** Prior probabilities of students' performance (SP) outcome interval.

	Periodic intervals of SP	Prior probability
1	0.1 ≤ SP ≤ 0.3	0
2	0.4 ≤ SP ≤ 0.6	0.00016
3	0.7 ≤ SP ≤ 0.9	0
4	1 ≤ SP ≤ 1.2	0.0072
5	1.3 ≤ SP ≤ 1.5	0
6	1.6 ≤ SP ≤ 1.8	0
7	1.9 ≤ SP ≤ 2.1	0.015
8	2.2 ≤ SP ≤ 2.4	0
9	2.5 ≤ SP ≤ 2.7	0
10	2.8 ≤ SP ≤ 3	0.0229
11	3.1 ≤ SP ≤ 3.3	0
12	3.4 ≤ SP ≤ 3.6	0.0458
13	3.7 ≤ SP ≤ 3.9	0.00286
14	4 ≤ SP ≤ 4.2	0.0315
15	4.3 ≤ SP ≤ 4.5	0.00573
16	4.6 ≤ SP ≤ 4.8	0
17	4.9 ≤ SP ≤ 5.1	0.0889
18	5.2 ≤ SP ≤ 5.4	0.0427
19	5.5 ≤ SP ≤ 5.7	0.00899
20	5.8 ≤ SP ≤ 6	0.12
21	6.1 ≤ SP ≤ 6.3	0.015
22	6.4 ≤SP ≤ 6.6	0.006
23	6.7 ≤ SP ≤ 6.9	0.009
24	7 ≤ SP ≤ 7.2	0.07429
25	7.3 ≤SP ≤ 7.5	0.0687
26	7.6 ≤ SP ≤ 7.8	0.0686
27	7.9 ≤ SP ≤ 8.1	0.1343
28	8.2 ≤SP ≤ 8.4	0.03143
29	8.5 ≤SP ≤ 8.7	0.06573
30	8.8 ≤ SP ≤ 9	0.115
31	9.1 ≤ SP ≤ 9.3	0.0315
32	9.4 ≤ SP ≤ 9.6	0.013
33	9.7 ≤ SP ≤ 9.9	0
34	9.9 ≤ SP ≤ 10	0.0088

**Table 3:** IMFS performance.

Partitions of students' performance outcome	IMFS precision	Values as recall	IMFS performance as *F*1 score	Specific accuracy measure
*P*1	0.709	0.782	0.7051	0.759
*P*2	0.733	0.797	0.7146	0.747
*P*3	0.708	0.789	0.7983	0.793
*P*4	0.794	0.778	0.7090	0.707
*P*5	0.723	0.787	0.7947	0.747

**Table 4:** Comparison with prior studies.

Features	Proposed IMFS	Prior study [50]	Prior study [51]	Prior study [52]
Quantization of students' performance	0 to 10	Not mentioned	Game score	LMS assignment

Frustration severity	Yes	No	No	No

Different levels of severity	4 levels	No	No	No

Quantization of students' performance periodic intervals	34	No	No	At-risk, failing, and excellent students

Prior probabilities as a coefficient	34 prior probabilities (like weights of a mathematical model) using Bayesian inference method	Markov property and attention mechanism	Hidden Markov model	No

Estimating students' performance with respect to frustration severity levels	Yes	No	No	No

Iterative refinement of students' performance probability	Prior probabilities are replaced by posterior probability. Further posterior is used as a prior and so on.	Bidirectional LSTM	No	No

Major characteristics	Quantization of students' performance, level of severity, periodic intervals [33], iterative estimation of performance outcome probability, and refinement of probability (memorize previous probability)	Exercise-enhanced recurrent neural network, bidirectional LSTM, and exercise-aware knowledge tracing	Comparative analysis findings	Analysis of decision tree, Naive Bayes, logistic regression, multilayer perceptron, and SVM on the bases of student performance prediction

Scalability	Number of performance outcome and periodic intervals are directly proportional with DSFN accuracy	Not explained	Not explained	Not explained

Proposed algorithm	Yes	No	No	No

Evaluation with number of accuracy measures	4	2	1	1

**Table 5:** List of abbreviations.

S.No	Abbreviations	Definitions
1	MOOCs	Massive Open Online Courses
2	IMFS	Iterative model of frustration severity
3	SP	Students' performance

## Data Availability

The data used to support the findings of this study are available from the corresponding author upon reasonable request.
